# Cloning Method for Stress-Resistant Gene of *Conringia planisiliqua* under Drought Stress

**DOI:** 10.1155/2021/3517002

**Published:** 2021-06-15

**Authors:** Yanfei Zhu, Yanying Qu, Melkamu Teshome Ayana

**Affiliations:** ^1^College of Agronomy, Xinjiang Agricultural University, Urumqi 830052, China; ^2^Department of Hydraulic and Water Resources Engineering, Arba Minch University, Arba Minch, Ethiopia

## Abstract

The low temperature, drought, high salt, and other environments influence crop production and development directly, so the gene cloning method has become an effective biological means. In order to effectively improve the cloning effect, a gene cloning method for *Conringia planisiliqua* based on mRNA differential display technology was proposed. Based on mRNA differential display technology, the gene of *Conringia planisiliqua* was transcribed. The present study expects gene cloning to be better than the traditional method. This will lay the basis for gene cloning and functional verification of the transcription and disease-resistant proteins in *Conringia planisiliqua*. According to homologous identification results, the homologous drought-resistant genes were determined and screened. The data of *Conringia planisiliqua* in the existing biological database were used to extract ESTs data of *Conringia planisiliqua*. Then, the heating environment was established and the concept of integral function was introduced to express the influence of growth environment of different genomes. The mass, momentum, energy, and turbulent flow situation of stress-resistant gene of *Conringia planisiliqua* during the growth were satisfied. Finally, the data search was carried out in the NCBI database and gene cloning was achieved by ESTs data sequence. Experimental results show that the proposed method can effectively reduce the gene data fitting and improve the quantity of gene fragments cloned in a cycle, so the overall cloning effect is better.

## 1. Introduction

Low temperature, drought, and saline-alkali conditions affect the yield and quality of crops seriously [1]. How to solve the crop yield reduction caused by these adverse conditions and make use of land resources, water resource is a major issue related to agricultural production. With the rapid development of molecular biology and the maturity of genetic engineering technology, improving the stress resistance of crops through genetic engineering is an effective way to improve crop yield [2]. How to use the resource of stress-resistant genes and find “key genes” from a large number of genes related to osmotic stress is an important precondition for plant osmotic stress genetic engineering. Because the stress resistance of plant is a complex quantitative character and it is also the result of multiple regulatory mechanisms, the transgenic plants with a single functional gene have no significant effect on resistance to osmotic stress [3]. In contrast, the transcription factor gene can regulate the expression of a series of downstream genes by combining with *cis*-acting elements, so as to achieve the cloning of stress-resistant genes. It is necessary to search for the transcription factors that play an important role in the process of stress resistance and then apply them to stress-resistant gene engineering. Thus, the ideal effect can be achieved by gene cloning [4].

*Conringia planisiliqua* belongs to the cruciferous *Conringia*, which is an ephemeral plant in early spring. *Conringia* contains eight species, and there is only one species in Xinjiang and Tibet [5]. It is a cruciferous herb. The height is 30–60 cm. The lower part is covered with single hairs and the upper part is glabrous. It is unbranched [6]. The seed is dark brown and short. The length is about 1.5 mm. It has a narrow edge and heavy hilum colour. The flower season is from May to June. It grows on the hillside of low mountain belt and dry riverbed, with an altitude of 900 m–1000 m. At present, the researches on ephemeral plants are mainly focused on population classification and seed biology. *Conringia planisiliqua* belongs to the tribe Brassicaceae in the system. Some researchers find that the chromosome number of *Conringia planisiliqua* is seven. But the researches on its internal genetic resources mining are not enough. In recent years, PEG6000 is used to simulate drought stress on six ephemeral plants, including *Conringia planisiliqua*. We can see that *Conringia planisiliqua* has a strong ability of drought resistance [7]. Some experts have cloned the CpHRD transcription factor gene of *Conringia* by homologous gene cloning technology and transformed the tobacco. The identification of related physiological indexes of drought resistance shows that the ability of drought resistance of transgenic tobacco with the CpHRD gene is significantly improved [8].

DDRT-PCR technology which was proposed by Japanese biological scientists in 2016 is widely applied in various fields of biotechnology, such as agriculture, plants, animals, medicine, and fungi, involving the gene induction and expression, heterosis mechanism, stress resistance, development molecular mechanism, gene cloning, and so on. In addition, this technology has successfully isolated hundreds of genes [9]. At present, there are few reports on the isolation and utilization of drought resistance genes in *Conringia*. In order to fully explore and utilize its drought resistance gene resource, it is necessary to research the mechanism of drought resistance mechanism from the molecular level. Therefore, this research uses mRNA differential display technology to select genes related to drought resistance of *Conringia*. Meanwhile, mRNA differential display technology is used to separate and recover the differentially expressed genes of *Conringia* under different conditions, then sequence them after the second PCR, and analyze their homology. In addition, the electronic homology cloning method is used to determine the DREB transcription genes of *Conringia* and find the core fragment of the drought-tolerance gene, so as to clone the gene under drought stress. It provides some candidate genes for further cloning of full-length drought-resistant genes and the breeding for stress resistance.

## 2. Methodology

### 2.1. Screening of Drought-Resistant Genes of *Conringia planisiliqua* Based on mRNA Differential Display Technology

#### 2.1.1. Gene Transcription and Homology Identification of Different Fragments

*Conringia planisiliqua* is a special short-lived plant in Xinjiang. This kind of plant lives in arid desert and gravel edge for a long time. In the long-term evolution, it adapts to the arid environment. There is a lack of understanding of the mechanism of stress resistance [10, 11]. The drought-resistant genes are screened by mRNA differential display. The seeds come from the plant teaching and research section of Xinjiang Agricultural University, and the seeds are planted and harvested in this laboratory [12]. First of all, the seeds were seeded in vermiculite, pearlite, and soil. The proportion is 1 : 2 : 3. They were cultured in the culture room with temperature of 23–25°C and light of 4000lx. After they grew to 3-4 weeks and there are 5–8 leaves, they were irrigated with 20% PEG6000. Then, drought stress treatment and NaCI-simulated salt stress treatment were simulated, and then seedling leaves after 0 h, 3 h, 6 h, 9 h, 12 h, and 24 h stress were collected [13]. After quick-freezing process with liquid nitrogen, they were stored in a refrigerator at 70°C. After that, RNA was extracted and purified with Trizol plant extraction kit of Tiangen, based on the instructions [14]. DNA was removed from RNA by DNase I kit. Moreover, 1.2% agarose gel electrophoresis was used to detect the quality of RNA. The reverse transcription kit and instructions were adopted. The 2 *μ*g RNA with four anchored primers is reverse transcribed to the first-strand cDNA (see Table 1).

After diluting the reverse transcript products for 5 times, we adopt 2 *μ*L template cDNA. Eighty pairs of PCR amplification primers are composed of four anchored primers and twenty random primers. The reaction system is 20 p*μ*L, including 10 × ExTaq Buffer 2 *μ*L, 2.5 mmol/L dNTP1L, 10 mmol/L anchor primer 1 *μ*L, and 10 mmol/L anchor primer 1 *μ*L. The 6% denatured polyacrylamide gel is used to test, and then they are photographed and recorded after colour reaction (see Table 2).

According to Table 2, the homology of different fragments is determined. The carrier sequence is removed by DNAMAN software (version 5.2; Lynnon Biosoft), and then the homology of different fragments is compared and analyzed by BLASTn software on the NCBI website. The closest sequence is used to annotate the biological function. The gene expression of drought and salt treatment is DF-2, DF-6, and DF-14 [15].

7500 Fast Real-Time PCR System is adopted. SYBR Green I fluorescent dye method was used to detect the gene transcription and expression levels of *Conringia planisiliqua* seedlings treated with 20% PEG6000 and 200 mm NaCI in different time periods.

#### 2.1.2. Filtering Operation

According to the results of RNA electrophoresis detection, the ratio of brightness display can be determined. After that, the detection results of UV spectrophotometer are recorded, and all records are applied to subsequent analysis (see Figure 1).

The results show that, in eighty primer combinations, the differential bands amplified by the primer pair composed of anchor primers have the best effect. The bands with increased or decreased expression are selected to retrieve and sequence, so that eighteen different bands with good reproducibility are obtained. The size of the band is basically 150–300 by, in which the size of the band is 414 bp and 559 bp. The average length of the bands is 231 bp. There are eighteen fragments with better specificity in secondary amplification. There are eighteen fragments based on the cloning sequencing (see Figure 2).

According to the results of electrophoresis detection, the sequence similarity is compared. Generally, the categories are as follows:

Based on similarity comparison, they can be divided into the following categories:

1. Three hypothetical protein-related fragments, hypothetical disease-resistance protein DF-1 of *Brassica* cabbage and hypothetical protein of mountain hollyhock, DF-3 and DF-4 [16].
2. Seven basic metabolism fragments, including receptor-like protein kinase 37 with a large content of cysteine, DF-5, cabbage vascular bundle protein DF-6, protein curvature of chloroplast thylakoid in *Brassica campestris* 1A, DF-7. *Arabidopsis* amino acid permeable enzyme1 mRNADF-8, *Brassica campestris* amino acid permeable enzyme 1, F-90 *Arabidopsis* peptidyl prolyl cistrans isomerase CYP63-like family protein mRNA, DF-16, and *Brassica napus* rich in glutamic acid cell wall structural protein with molecular level 120.
3. Three disease-resistant proteins, radish specific albumin 5, DF-2, *Arabidopsis* AMC7DF-10, and *Brassica napus* MLO-like protein 12, DF-110.
4. Two unknown proteins, DF-17 and DF-180.
5. Two photoperiod-related proteins (CCAL and DF-13) in *Arabidopsis*. GATA transcription factor 13 is assumed in *Camelina*, DF-15. The GATA transcription factor 13 assumed in *Camelina* may play a regulatory role in light response genes.
6. One transcription factor, DF-14, similar fragments of *Arabidopsis thaliana* alfin-like protein. The details are shown in Table 3.

The research shows that the expression of DF-2 and DF-14 was raised dynamically with time under PEG6000 stress treatment. The expression level of DF-2 reached the highest value at 9 h and DF-14 reached the highest value at 6 h. DF-6 expression came down by the influence of PE 66000. Under the salt stress, DF-2 and DF-14 were upregulated dynamically with time, and the expression of them reached the highest level at 24 h. DF-6 was the highest at 3 h, and then it was lower than the contrast. The results show that the response speed of DF-2 and DF-14 to the salt stress was slower than that of DF-6. Therefore, the expression of DF-2, DF-6, and DF-14 is induced by drought and salt.

According to statistical results, the final gene function and proportion are determined as shown in Figure 3.

According to the gene results shown in Figure 3, based on the relationship between drought stress and salt stress, the fluorescence quantitation is used to determine the overall format of the selected gene segment. See Figure 4.

According to the screened genes, we can see that the fragments of genes are generally small, so it is difficult to research the gene further. It is necessary to select the longer fragments with unknown functions for further research. The random combination of the anchor primer Oligo (dT) *M*_2_ produced the most differential bands, which are recycled from thirty selected strips. Eighteen bands are cloned and sequenced. The positive rate is 60%.

In terms of the discovered gene classification, the proportion of hypothetical protein was maximum, 38.89%. Next is the proportion of transcription factors and disease-resistant protein, 16.67%. The proportion of unknown protein is the same as the proportion of photoperiodic protein, 11.11%. The proportion of basic metabolism is 5.56%. This result also shows that related protein kinase, vascular bundle protein, photosynthesis, amino acid permeable enzyme, *cis*-trans isomerase, cell wall structural protein, and transcription factor participate in response to the drought stress. However, the photoperiod and disease-resistance proteins also respond, which was rarely found at present. The stress resistance mechanism of plants is the intercrossing stress. Some genes can participate in the biological and abiotic stress of plants. There are many related researches on the genes of basic metabolism, so it is necessary to research the disease-resistant protein, hypothetical protein, unknown protein, and transcription factor further.

### 2.2. ESTs Data Acquisition of *Conringia planisiliqua*

All EST data of wild soybean are downloaded from the EST database (dbEST) of NCBI, and there are 18511 data in total. The Linux sequence analysis platform constructed in this research is adopted and the above gene data is used to remove redundant data. There are 9983 unigene data in total. Contigs of 9983 wild *Conringia* are compared with 61036 probe groups contained in A Metrix soyabean gene expression analysis chip by BLASTn. The signal changes of chip probe groups are used to annotate the expression changes of corresponding *Conringia* at the early stage of different permeation stress (1 h). The upregulated expression is selected at least stress. Meanwhile, the annotation information contains contigs with kinase as the material for further study. For the expression level, eighteen protein kinase ESTs are upregulated under 40°C stress. Twenty protein kinase ESTs are upregulated under NaCI stress. Twenty-seven protein kinase ESTs are upregulated under PEG stress. The nonredundant protein kinase EST based on the partial expression of *Conringia* is shown in Table 4.

TreEMBL/SWISS-PROT database and GenBank database are used to analyze all kinase contigs by BLAST, and the related literature about the subject is consulted to further predict the function of ESTs. The protein kinase ESTs related to stress signal transduction are selected. In order to ensure the balance of *Conringia* data and the normality of EST data, it is necessary to design the coupling model with the help of solar indoor light and environment distribution.

The solar active heating room is adopted in the design, and its core conditions are as follows.

Firstly, the air in solar active heating room adopted for *Conringia* data extraction is the incompressible air, which conforms to BOUTER standard. Secondly, the indoor air environment has the feature of steady-state flow and turbulent flow. Thirdly, this research ignores the thermal radiation between solid walls. Fourthly, there is no obvious air leakage in the designed heating room. According to the above assumptions and nonredundant protein kinase EST data, the turbulence flow equation is added to the environmental construction.

In order to extract the complete gene data, the concept of integral function should be introduced into the extraction environment of the designed heating room to represent the influence of different genome growth environment, so as to meet the quality, momentum, energy, and turbulence situation in the growth process of the stress-resistant gene of *Conringia*. The key point is the gaseous phase of gene distribution. In the following equations, *p* and *q* represent the volume fractions, respectively. Taking the comparison of *q* and particle phase in the greenhouse as an example, it should satisfy the conservation equation of growth mass:

(1) $$\begin{array}{c} \frac{\partial }{\partial t}\left(\alpha_{q}\rho_{q}{\overset{⟶}{v}}_{q}\right)+\nabla \left(\alpha_{q}\rho_{q}{\overset{⟶}{v}}_{q}{\overset{⟶}{v}}_{q}\right)=-\alpha_{q}\nabla P\\ \nabla •\tau_{q}+\alpha_{q}\rho_{q}\overset{⟶}{g}+\sum_{p=1}^{n}R+mv-m\overset{⟶}{v}+\\ \left(F_{q}+F_{\text{lift},q}\right). \end{array}$$

In equation (1), ${\overset{⟶}{v}}_{q}$ denotes the phase velocity of particle in the current gene. *α*_*q*_ denotes the mass transfer process indoor. *ρ*_*q*_ denotes the reverse mass transfer process. *q* is compared with the particle phase of *Conringia*. Let it satisfy the equation of conservation of momentum:

(2) $$\begin{array}{c} \frac{\partial }{\partial t}\left(\alpha_{q}\rho_{q}{\overset{⟶}{v}}_{q}\right)+\nabla \left(\alpha_{q}\rho_{q}{\overset{⟶}{v}}_{q}{\overset{⟶}{v}}_{q}\right)=\alpha_{q}\nabla P\\ \nabla •\tau_{q}+\alpha_{q}\rho_{q}\overset{⟶}{g}+\sum_{p=1}^{n}R+mv-m\overset{⟶}{v}\\ +\left(F_{q}+F_{\text{lift},q}+F_{vm,q}\right). \end{array}$$

In equations (1) and (2), *τ*_*q*_ is the actual expansion of stress and strain of *Conringia*. The specific calculation is

(3) $$\begin{array}{c} \tau_{q}=\frac{\alpha_{q}\mu_{q}\left(\nabla v_{q}+\nabla v_{q}^{T}\right)}{\alpha_{q}\left(\lambda_{q}-\left(2/3\right)\right)}\mu_{q}. \end{array}$$

In equations (2) and (3), *μ*_*q*_ and *λ*_*q*_ denote the actual maximum shear viscosity and average crimp volume viscosity of gene particle phase in the current extraction environment. *F*_*q*_ denotes the external volume stress of indoor air particle phase. *F*_lift,*q*_ denotes the maximum lifting stress of particle phase. *F*_*vm*,*q*_ denotes the actual lubrication force of gene phase wall. *v*_*q*_^*T*^ denotes the force existing in the current indoor particle phases. At this time, *T* is the actual turbulent diffusion force.

*q* term is used to compare the particle phase in greenhouse. Let it meet the energy conservation equation.

(4) $$\begin{array}{c} \frac{\partial }{\partial t}\left(\alpha_{q}\rho_{q}{\overset{⟶}{v}}_{q}\right)+\nabla \left(\alpha_{q}\rho_{q}{\overset{⟶}{v}}_{q}h_{q}\right)\\ =\alpha_{q}\frac{\partial p_{q}}{\partial t}+\alpha_{q}\rho_{q}\overset{⟶}{g}+Sq+\left(Qpq+m_{pq}h_{pq}-m_{qp}h_{qp}\right). \end{array}$$

In equation (4), *h*_*pq*_ denotes the maximum specific heat enthalpy of the current particle phase. *S*_*q*_ denotes the hot-gas source generated by drought stress factors. *Q*_*pq*_ represents the intensity conversion between gas phase and particle phase in the current environment. *h*_*qp*_ denotes the highest enthalpy between gas phase and particle phase.

Different energy equations are introduced into the general turbulence formula to calculate the relationship variables. The general form is as follows:

(5) $$\begin{array}{c} \text{div}\left(\rho v\phi \right)=\text{div}\left(F\phi \text{grad}\phi \right)+S\phi . \end{array}$$

In equation (5), div(*Fϕ*grad*ϕ*) is the diffusion term of current turbulent, and *Sϕ* denotes the generalized source term.

The boundary condition of *Conringia* ESTs data calculation: term value should be added to the actual coupling point of the current indoor convection boundary. Because the drought environment will bring the radiation heat source, the constant heat flow is used to represent the current radiation. The actual lighting condition and air supply temperature condition are added, so as to adjust the corresponding pressure of indoor air return outlet to the initial value, 0. In addition, additional boundary conditions are not needed to be added to the interface between air fluid and nonfluid in the drought environment simulation. The energy relationship in the current gene coupling process is compared numerically. Under the action of solar radiation, the radiation dispersion will be generated, so it is necessary to simulate based on the above coupling environment.

(6) dupdt=FDup−ug,FD=18μgρlDp2CDRed,

(7) $$\begin{array}{c} \frac{\text{d}x}{d_{t}}=u_{p},\frac{\text{d}r}{d_{t}}=v_{p}. \end{array}$$

Equation (6) is the equation of particle phase motion under drought stress. Equation (7) is the orbital equation of particle phase.

During the discrete phase orbit simulation, the current greenhouse structure can be regarded as a bisymmetry structure of rotating axis, so the calculation of control equation is also carried out in the way of two-dimensional symmetry. In this design, N-S equation is used to simulate the discrete phase orbit. The equation is as follows:

(8) $$\begin{array}{c} \frac{\partial U}{\partial t}+\frac{\partial F}{\partial x}+\frac{\partial G}{\partial y}+H=0. \end{array}$$

In equations (6)–(8),

(9) $$\begin{array}{c} U=r\left(\rho ,\rho u,\rho E\right)T,\\ F=r{\left(\rho u,\rho u^{2}-T_{xx},\rho uv-T_{xr},\rho Eu-T_{xx}u\right)}^{T},\\ G=r{\left(\rho_{v},\rho_{uv}-T_{rx},\rho v^{2}-T_{rr}\right)}^{T},\\ H={\left(0,0,\tau_{\theta \theta },0\right)}^{T},E=\left(\gamma -1\right)\frac{p}{\rho }+\frac{1}{2}\left(u^{2}+v^{2}\right),\\ T_{xx}=-p-\frac{2}{3}\mu \left(\frac{\partial v}{\partial r}+\frac{v}{r}\right)+\frac{4}{3}\mu \frac{\partial u}{\partial x},\\ T_{rr}=-p-\frac{2}{3}\mu \left(\frac{\partial u}{\partial x}+\frac{v}{r}\right)+\frac{4}{3}\mu \frac{\partial v}{\partial r},\\ \tau_{\theta \theta }=-p-\frac{2}{3}\mu \left(\frac{\partial u}{\partial x}+\frac{\partial v}{\partial r}\right)+\frac{4}{3}\mu \frac{v}{r},\\ T_{rx}=\mu \left(\frac{\partial u}{\partial r}+\frac{\partial v}{\partial x}\right),\\ q_{x}=-k_{\text{eff}}\left(\frac{\partial T}{\partial x}\right),\\ q^{r}=-k_{\text{eff}}\left(\frac{\partial T}{\partial r}\right),\\ k_{\text{eff}}=k_{L}+k_{T},\\ \mu =\mu_{L}+\mu_{T}, \end{array}$$

where *T* denotes time; *μ* denotes the current viscosity coefficient; *γ* denotes the thermal energy ratio in the current environment; *k* denotes the thermal conductivity in the current room; *x* is the axial coordinate of discrete phases; *r* denotes the current radial coordinate; *ρ* denotes the environmental thermal imagery density; *u* denotes the axial speed; *v*represents the radial speed; *p* represents the environmental pressure; *E* is the internal energy under the action.

Finally, ESTs data are calculated. The definition of *Conringia* ESTs is as follows:

(10) $$\begin{array}{c} HL_{n}=KF\left(t-t_{w}\right)\varepsilon . \end{array}$$

In equation (10), *F* is the area unit of the enclosure is based on square meters; *K* is the heat conduction coefficient of the current drought simulation structure. Generally, the unit is W/m^2^ °C. *t* is the designed temperature. *t*_*w*_ is the actual outdoor temperature in the current heating. *ε* is the current heat load coefficient ratio.

### 2.3. Achievement of Stress-Resistant Gene Cloning of *Conringia planisiliqua*

The stress-resistant genes of *Conringia* extracted above are transcribed into the factor gene library. Because the gene sequence of DREB transcription factor is the seed, *Glycine soja* is regarded as the restriction word according to ESTs data. The data is searched in the database on NCBI to obtain relevant EST sequence. The sequence of EST was spliced by Contig Express splicing software, and then contigs are compared by BLASTn on NCBI. According to the comparison results, the contigs that may be DREB transcription factor genes are selected to predict the full length and ORF. According to the contig 5 sequence, a pair of primers is designed to verify the accuracy of the splicing result. The primers are also designed at both ends of the extended genome sequence contigs. The target fragments are amplified from RNA of *Conringia* by RT-PCR, and then they are cloned and sequenced. The sequence of primer design is as shown in Figure 5.

Fill in *Bacillus coli* for transformation. The steps are as follows:

 
*Step 1*. In the connection product, we add equal volume of IM NaCl.
 
*Step 2*. Add the DNA to be transformed into 100 *μ*L of competent cells. Then, mix it gently and place it on ice for 30 min.
 
*Step 3*. Thermal excitation is performed at 42°C for 90 s, then put it back in the ice to cool for 1–2 min, after that, the thermal excitation is performed at 42°C for 20 s, then put it back in the ice to cool for 1–2 min 1-2 min, and add 500∼600 *μ*L fluid LB, 370°C, 180 rpm, shaking culture for 45 min.
 
*Step 4*. Transfer the transformed competent cells to LB solid medium containing antibiotics (37°C preheating). Absorb 100 L bacterial solution, and use a sterile glass rod with elbow to coat the entire plate with bacterial solution.
 
*Step 5*. Invert the experimental plate and culture at 37°C for 12–16 h; then the bacterial colony appears.

DNA in tissues is extracted by the method of alkaline lysis procedure. The specific steps are as follows:

- Single colonies are selected and inoculated into Sml *LB* liquid medium containing corresponding antibiotics and cultured overnight at 37°C and 200 rpm.
- Pour 1.5 m1 bacterial solution into the centrifuge tube, 12000 rpm, centrifuge for 30 s, and remove the supernatant.
- Add 100 *μ*L cold solution I and the oscillates to make the bacteria resuspended.
- Add 200 *μ*L new solution II, mix it upside down, and ice bath is performed for Smin0.
- Add 150 *μ*L cold solution III, reverse and mix it well, and then take an ice bath of Smin0.
- Centrifuge for *s* min at 12000 rpm and 40°C and move the supernatant to a new pipe.
- Add solution of equal volume and the proportion of phenol and chloroform is 1 : 1, and shake and mix them. With the speed of 12000 rpm, centrifuge it for Smin. Then, the supernatant is moved to a new pipe.
- Add 2 times the volume of 95% cold ethanol, mix it upside down, and place it at room temperature for 30 min.
- Centrifuge for *S_min_* at 10000 rpm and 4°C.
- Supernatant is removed to add 1 ml 70% ethyl alcohol and clean.
- Pour out the ethanol and dry it in the air.
- Dissolve it in 20 *μ*L TE, detect by 0.8% agarose gel electrophoresis (SV/cm voltage), and store it at −20°C.

Finally, PCR identification and positive clone were carried out.

PCR reaction system is shown in Table 5, and PCR reaction condition is shown in Table 6.

Single colony was used as a template. PCR was used to complete the detection. Finally, the positive clone was completed.

## 3. Experimental Inquiry

In order to verify that the above methods can effectively improve the cloning effect, the comparative verification was carried out in the laboratory environment. Based on statistics division, the data of this experiment were tested by SAS8.1 software. According to Duncan, the significant difference was tested.

According to the previous research results in laboratory, an EST sequence was isolated from HarvEST database. Since the genomic database of Conringia planisiliqua was not published, RACE (Rapid amplification of cDNA ends) technology was used to amplify the third and fifth end of the sequence. The fragments with the length of 254 and 153 Kbp were obtained from 3'-end and 5'-end RACE PCR, respectively. Then, these two sequences were spliced with the original EST sequence to form a complete gene sequence that was verified by PCR. The total length of cDNA sequence is 428 by, including 141 by ORF and encoding forty-six amino acids. The amplified genome sequence was consistent with the full length of its cDNA sequence, so that the sequence contained only one exon without intron structure. When analyzing the possible domain of protein, the results show that this protein does not contain any known conserved domain, except for a repetitive structure composed of thirteen amino acids with low complexity.

ExPASY predicted that the relative molecular weight and isoelectric point of this protein were 4.94 kD and 3.760, respectively. Moreover, this sequence was imported into NCBI online database for BLAST analysis. We can see that this gene sequence is basically the same as that of an unidentified site geneLOC102619665 CXR 369802 in *Conringia planisiliqua*, and it also has about 77% sequence similarity with potential DNA binding protein CsV03-3 CEF175925. However, the homologous gene was not found in other species. The result of _L shows that the sequence was unique in citrus, so it is named FcSISP. Taking FcSISP as the data sample, we analyzed and compared the cloning effect of the designed gene cloning method. The statistical results are shown in Figures 6 and 7.

According to the above comparison result, for the cloning target of gene combination chain generated in the current laboratory, the designed cloning method is compared with TSA cloning method, multicomputer cloning method, and over-the-horizon cloning method. We can see that the designed cloning method has the lowest fitting index and more gene fragments per unit cycle. Thus, the effectiveness of the proposed method can be proved.

## 4. Conclusions

The analysis on the mRNA difference under the drought stress of *Conringia planisiliqua* of *Conringia* of Cruciferous ephemeral plant shows that eighteen gene segments induced or inhibited by drought are obtained. The proportion of hypothetical protein is 38.89%. The proportion of disease-resistant protein is 16.67%. The proportion of unknown protein is 11.11%. The proportion of photoperiod protein is 11.11%. The proportion of basic metabolism is 5.56%. The proportion of transcription factors is 16.67%. On this basis, the result of gene cloning is better than that of the traditional method, which lays a foundation for gene cloning and functional verification of transcription factors, basic metabolism, and disease-resistant proteins in *Conringia planisiliqua*. This also provides a theoretical basis for the exploration of wild stress-resistant plant resource. Experimental results show that the proposed method can effectively reduce the gene data fitting and improve the quantity of gene fragments cloned in a cycle, so the overall cloning effect is better.

## Figures and Tables

**Figure 1:** Total RNA electrophoresis of *Conringia planisiliqua*.

**Figure 2:** Detection results of 6% electrophoresis of partial CDNA differential bands.

**Figure 3:** Function classification and proportion.

**Figure 4:** DF-2 DF-6 DF-14 fluorescence expression.

**Figure 5:** Schematic diagram of primer design.

**Figure 6:** Comparison of the fitting index of multiple gene cloning methods.

**Figure 7:** Comparison of maximum data storage of the system.

**Table 1:** Anchor primers of RNA differential display.

The name of the primer	Primer sequence 5–3
M1	ACGACTCACTATAGGGTTTVA
M2	ACGACTCACTATAGGGTTTVG
M3	ACGACTCACTATAGGGTTTVG
M4	ACGACTCACTATAGGGTTTVT

**Table 2:** Random primers for mRNA differential display.

The name of the primer	Primer sequence 5–3
R1	ACGACTCACTATAGGGTTTVG
R2	ACGACTCACTATAGGGTTTVG
R3	ACGACTCACTATAGGGTTTVG
R4	ACGACTCACTATAGGGTTTVT
R5	ACGACTCACTATAGGGTTTVT
R6	ACGACTCACTATAGGGTTTVG
R7	ACGACTCACTATAGGGTTTVC
R8	ACGACTCACTATAGGGTTTVG
R9	ACGACTCACTATAGGGTTTVA
R10	ACGACTCACTATAGGGTTTVG
R11	ACGACTCACTATAGGGTTTVA
R12	ACGACTCACTATAGGGTTTVH
R13	ACGACTCACTATAGGGTTTVG
R14	ACGACTCACTATAGGGTTTVY
R15	ACGACTCACTATAGGGTTTVG
R16	ACGACTCACTATAGGGTTTVT
R17	ACGACTCACTATAGGGTTTVA
R18	ACGACTCACTATAGGGTTTVG
R19	ACGACTCACTATAGGGTTTVG
R20	ACGACTCACTATAGGGTTTVG
R21	ACGACTCACTATAGGGTTTVG
R22	ACGACTCACTATAGGGTTTVG
R23	ACGACTCACTATAGGGTTTVY
R24	ACGACTCACTATAGGGTTTVT

**Table 3:** Comparison of DFs sequence and BLAST sequence in NCBI accounting sequence database.

Name of the sequence	The length of the function	Match login number	*E* value
DF-1	Hypothetical disease-resistance protein of *Brassica* cabbage	AB751520	6*E−*27
DF-2	Radish specific albumin 5	AB751521	1*E−*64
DF-3	Hypothetical protein of mountain hollyhock	AB751522	7*E−*48
DF-4	*Camelina*, receptor-like protein kinase 37 with a large content of cysteine	AB751523	5*E−*25
DF-5	Cabbage vascular bundle protein	AB751524	4*E−*170
DF-6	Protein curvature of chloroplast thylakoid in *Brassica campestris* 19	AB751525	6*E−*66
DF-7	*Arabidopsis* amino acid permeable enzyme 1 mRN A	AB751526	6*E−*52
DF-8	*Brassica* cabbage amino acid permease 1	AB751527	3*E−*60
DF-9	*Arabidopsis* metacaspase 7	AB751528	1*E−*2
DF-10	*Brassica napus* MLO-like protein 12	AB751529	8*E−*17
DF-11	*Brassica napus* glutamic acid rich cell wall structural protein 1	AB7515210	6*E−*27
DF-12	mRN a of *Arabidopsis* CCAl protein	AB7515211	6*E−*30
DF-13	mRNA of *Arabidopsis thaliana* alfin-like protein	AB7515212	5*E−*42
DF-14	*Camelina sativa* hypothesis GATYA transcription factor 13	AB7515213	4*E−*2
DF-15	*Arabidopsis* peptidyl-prolyl *cis*-trans isomerase CYP63-like family protein mRNA	AB7515214	3*E−*87
DF-16	Hypothetical protein of mountain hollyhock	AB7515215	2*E−*28
DF-17	Unknown characteristic protein ycf39-like	AB7515216	6*E−*20
DF-18	*Brassica napus* unknown protein	AB7515217	1*E−*14

**Table 4:** Nonredundant protein kinase EST based on partial expression of *Conringia*.

Unigene	Induced by	Probe number	Probe annotation
CL68076contig 1	PEG	GMA2544.1	Pyrophosphate-dependent phosphofructokinase

CL997contig 1	4 Celsius degrees	GMA4354.1	Glycine max cv prize protein kinase
	NaCL		
	PEG		

CL1185contig 6	4 Celsius degrees	GMA2214.1	Lectin-like protein kinase
	NaCL		
	PEG		

CL1235contig 5	4 Celsius degrees	GMA1934.1	Phosphoribulokinase
	NaCL		

CL145076contig 1	NaCL	GMA2054.1	Protein kinase
	PEG		

CL758contig 1	PEG	GMA1684.1	Phosphoglycerate kinase
	NaCL		
	4 degree Celsius		

CL755contig 1	PEG	GMA2204.1	Protein kinase
	4 degree Celsius		
	NaCL		

CL1230contig 4	PEG	GMA1364.1	HXK2 ARATH hexokinase 2
	NaCL		

CL 1238contig 1	PEG	GMA3784.1	Leucine-rich repeat transmembrane protein kinase 1
	4 degree Celsius		
	NaCL		

CL 1138contig 1	PEG	GMA2204.1	Glycine max choline kinase GmCK2pmRNA

CL 1285contig 1	PEG	GMA1934.1	Phosphoglycerate kinase
	NaCL		

**Table 5:** Parameters of PCR reaction system.

Deionized water	19.3 *μ*L
10 × PCR buffer	2.5 *μ*L
DNTP	2.0 *μ*L
P3	0.5 *μ*L
P5	0.5 *μ*L
The template	A single colony
RTaq enzyme	0.2 *μ*L
The total volume	25 *μ*L

**Table 6:** PCR parameters of reaction condition.

Predenaturation at 95 degrees Celsius	7 min
95 degree Celsius denaturation	30 s
Annealing at 55°C	30 s
Extension at 72°C	1 min 35 s
Extension at 72°C	7 min
The reaction ends at 4 degrees Celsius	

## Data Availability

The data used to support the findings of this study are available upon request.
